The article "An Empirical Analysis of an Optimized Pretrained Deep Learning Model for COVID-19 Diagnosis" was published in 2022. Journal: Comput Math Methods Med.

# An Empirical Analysis of an Optimized Pretrained Deep Learning Model for COVID-19 Diagnosis

**DOI:** 10.1155/2022/9771212

**Published:** 2022-07-27

**Authors:** S. K. B. Sangeetha, M. Sandeep Kumar, Deeba K, Hariharan Rajadurai, V. Maheshwari, Gemmachis Teshite Dalu

**Affiliations:** ^1^Department of Computer Science and Engineering, SRM Institute of Science and Technology, Chennai, India; ^2^School of Information Technology and Engineering, Vellore Institute of Technology, Vellore, Tamil Nadu, India; ^3^School of Computer Science and Applications, REVA University, Bangalore-560064, India; ^4^School of Computer Science and Engineering, Vellore Institute of Technology, Bhopal, India; ^5^Department of Software Engineering, College of Computing and Informatics, Haramaya University, POB 138, Dire Dawa, Ethiopia

## Abstract

As a result of the COVID-19 outbreak, which has put the world in an unprecedented predicament, thousands of people have died. Data from structured and unstructured sources are combined to create user-friendly platforms for clinicians and researchers in an integrated bioinformatics approach. The diagnosis and treatment of COVID-19 disease can be accelerated using AI-based platforms. In the battle against the virus, however, researchers and decision-makers must contend with an ever-increasing volume of data, referred to as “big data.” VGG19 and ResNet152V2 pretrained deep learning architectures were used in this study. With these datasets, we could train and fine-tune our model on lung ultrasound frames from healthy people as well as from patients with COVID-19 and pneumonia. In two separate experiments, we evaluated two different classes of predictive models: one against pneumonia and the other against non-COVID-19. COVID-19 can be detected and diagnosed accurately and efficiently using these models, according to the findings. Therefore, the use of these inexpensive and affordable deep learning methods should be considered as a reliable method for the diagnosis of COVID-19.

## 1. Introduction

The current Coronavirus 2019 (COVID-19) pandemic situation is a threat to humanity and also affects the entire global economy, as evidenced by the prevalence of infections and epidemics over the last 20 years. In 1960, the first coronaviruses were discovered [1]. To prevent the spread of the new coronavirus, health workers, governments, and the general public must work together. First-hand computed tomography (CT) images and clinical data are essential for clinical decision-making and for providing information that can deepen our understanding of the patterns of infection by the virus and provide systematic models for early diagnosis and timely medical interventions in the face of the global spread of COVID-19 [2, 3]. Open-access CT images and clinical symptoms from around the world are needed to help in the fight against COVID-19. Because we are working with CT slides as our input images, the problem with detecting COVID-19 is one of the image classifications [4, 5].

By using CT scan images, it is possible to identify COVID-19 cases, but their specificity is low. CT scans are more accurate in cases of COVID-19 but less accurate in cases of nonviral pneumonia as a result of this change. Chest CT scans are effective for detecting lung damage caused by COVID-19 [6, 7]. Although some drawbacks exist, it is still a viable option. There are patients whose CT results are normal at the onset of the illness that cannot be diagnosed with CT alone, which is contrary to WHO recommendations. CT scans may miss non-COVID-19 cases because of their low sensitivity [8–10]. To overcome the limitations of COVID-19 diagnostic tests, researchers have studied the use of deep learning (DL) in radiological image analysis. Large-scale research into DL algorithms, particularly CNN, was spurred by COVID-19. The use of DL techniques to examine CT scan images revealed that numerous attempts have been made to enhance these methods [11].

The ability of these methods to detect COVID-19-induced pulmonary lesions rests on their ability to extract and select features hidden within the images. The lack of DL equipment in all medical and diagnostic centres was one of the biggest drawbacks of DL algorithms after an improvement in COVID-19 diagnostic detection and diagnosis. Additional CT scans of the chest were necessary for many COVID-19 patients as well. For patients, radiation exposure during CT scans can lead to life-threatening health issues [12, 13]. Furthermore, a patient's virus could be spread to others through contaminated CT scan tunnels. Patients with COVID-19 can be detected, and infectious lung tissue can be extracted using DL's image feature extraction capabilities.

The main contributions of the work are as follows:

1. Data is collected for the purpose of developing an AI-based application that can identify and distinguish between different types of infection
2. Type of virus, type of bacterium, and type of fungus are all labelled and arranged in a hierarchy in the dataset
3. Data is gathered from public sources, as well as from hospitals and doctors, via indirect collection
4. Deep learning pretrained models VGG19 and ResNet152V2 are created for the real dataset and used for predicting three classes of outcomes: healthy, COVID-19-associated pneumonia, and COVID-19-associated pneumonia but without COVID-19

The remainder of the paper is organised as follows: system model is described in Section 3, experimental results and analysis are shown in Section 4, and the conclusion is provided in Section 5.

## 2. Literature Study

COVID-19 has wreaked havoc on the global economy. After starting in Wuhan, China, the COVID outbreak has now spread to various parts of the world. Machine learning (ML) can be used in a variety of ways, including text mining, spam detection, video recommendation, picture categorization, and multimedia idea retrieval [14]. Deep learning is a popular computer paradigm for machine learning, but it is also one of the most expensive. Deep learning has the ability to process enormous amounts of data, which is a significant advantage. CNNs are the most widely used deep learning algorithm, according to a recent study. In contrast to traditional fully connected networks, CNN algorithms use shared weights and local connections instead of global connections to fully exploit 2D input data formats like image signals [15].

In addition to posing a serious risk to human health, zoonotic diseases could have far-reaching consequences for the global economy. No nation can operate effectively as an island in today's global economy, as evidenced by the recent appearance of COVID-19. Public health and economic growth require a global perspective. It is imperative that all of the world's most populous countries participate in this effort. It is pointless to try and stop a pandemic after it has already spread to another country [16]. A lack of information and an overflow of noise and outliers limit its usefulness. Data is required for the training of an artificial intelligence system. Globally, there has been an increase in activity in this field. Despite the fact that this is encouraging, more research is required. Effective data management is required to reduce the epidemic's human and economic costs in addition to providing training data for AI models. When restrictions are eased, additional diagnostic testing will help to slow or even halt this epidemic, as well as reduce the economic harm that lockdowns cause [17].

In order to get a better sense of how many people are still infected but not showing any symptoms, they recommend conducting additional testing on a larger sample size. At this time, there is no way to estimate how many people have been affected. To make matters worse, it is estimated that 86% of all illnesses go unreported. If that is the case, the pandemic could resurface, delaying the economy's return to normalcy even longer. As a result, it is critical to address the knowledge gap regarding who is contagious [18, 19]. The 2019-nCoV condition should be identified and evaluated through the use of CT scans in individuals with first negative reverse transcription polymerase chain reaction (RT-PCR) or asymptomatic results. According to this hypothesis, patients who have asymptomatic or false-negative RT-PCR results may benefit from screening with early CT changes. Coronavirus infection needs to be found and treated as soon as possible. To prevent the development of acute respiratory distress syndrome (ARDS) in patients with pneumonia, corticosteroid therapy and other effective therapies should be considered. The faces and urine of patients with no symptoms or a positive test result should be thoroughly examined [20, 21].

Table 1 shows the comparison of some highlighted related works. In order to confirm positive patients and provide timely treatment, the primary goal is to improve COVID-19 diagnostic accuracy. Artificial intelligence (AI) requires data to be screened and relevant attributes to be calculated rather than the proper structure and unification required by traditional statistics. Using four different algorithms and artificial intelligence technologies, this study examines the three sets of data: the confirmed group, the unconfirmed group, and the total [25]. Artificial intelligence has become increasingly popular in the treatment of cancer patients as a result of our previous research. The accuracy of predictions and diagnoses can be improved by AI's ability to reduce human error in large-scale studies. COVID-19 detection data can be quickly mined for correlations between indicators, and a minimum correlation is sought in order to reduce the number of redundant indicators [26, 27]. The brief review seeks to outline and assess the reliability and efficacy of some of the most important AI-powered techniques for predicting COVID-19 spread [28].

Traditional statistical methods can be interpreted using traditional statistical methods because of the interpretability of screening indicators taken into account by the artificial intelligence method. There are still holes in the research because of the small sample size and the use of limited clinical data. There was no comparison to clinical trials in this study [29, 30]. In the future, we hope to verify and mine more accurate and effective detection models based on AI-based clinical diagnosis and prediction and provide decision support and aid for correct diagnosis and treatment of this condition through more comprehensive clinical data analysis. Additional deep learning models can be used to detect other medical issues, allowing the system to be widened. It is also possible to improve chest X-ray picture analysis by making changes to the algorithms that generate activation maps. The accuracy of a deep learning model can be greatly improved by using better datasets during training [31].

## 3. System Methodology

The layers of a CNN are designed to transform an image into an output that the model can comprehend. A feature map is generated using a convolutional layer, which applies a filter to the image and scans it one pixel at a time. The convolutional layer generates a large amount of data, so the pooling layer reduces the size of that data for storage. As a result of the inputs being fully connected, the outputs are flattened into a single vector. Applying weights based on feature analysis is done on fully connected layer inputs. Final probabilities generated by a fully connected output layer can be used to determine the class of an image. In order to find the optimal weights and activate only the most powerful and predictive neurons, an iterative forward and backward propagation process goes through all of the network training samples. Running through all of the training samples once forward and once backward is used to train the model [32]. Using forward propagation, we can determine the loss and cost functions for each labelled image by comparing the observed and predicted targets. Updating the weight and bias of each neuron using gradient descent prioritises the neurons with the highest predictive power until the optimal combination of activation is found for that neuron [33]. As more examples are fed into the model, it becomes more accurate at predicting the target, resulting in a smaller loss. Overall performance is determined by averaging the losses across all samples.  Figure 1 depicts the proposed deep learning framework for classification.

### 3.1. Optimized VGG19 Model

VGG19 is an advanced CNN with pretrained layers and a great understanding of what defines an image in terms of shape, color, and structure. VGG19 is very deep and has been trained on millions of diverse images with complex classification tasks.

### 3.2. Procedure

- Image direction should be reversed in order to include images that are similar to your target
- Use versions with and without blur
- Reduce image dimensionality by compressing spatial size and parameters with maximum pooling between layers
- Avoid overfitting by stopping early; if the model reaches its peak accuracy, it will stop looking for an even higher accuracy after a certain number of epochs
- To reduce the amount of time it takes to train, use fewer epochs
- Sigmoid and tanh activation functions are inefficient compared to rectified linear unit (ReLU), which only activates specific neurons
- Dropout can be used to reduce network computation by ignoring randomly selected neurons during training
- Avoid images with a lot of pixels because they do not help students learn much (224 by 224 pixels is the standard)

### 3.3. Optimized ResNet152V2 Model

ResNet152V2 is also used as feature extraction models. The models can train the input based on their pretrained initial weights. This approach accelerates the training and coverage to high accuracy.  Table 2 depicts the proposed layers for pretrained ResNet models.

Image scaling, reshaping, and array conversion are all part of the preprocessing. The same processing is applied to the test image. A collection of approximately 2000 images, both COVID and non-COVID, is suitable for use as software test images. The first step in the detection process is to improve the image quality in order to remove unwanted image detail, which is commonly referred to as image noise. Raw picture images have distortions. Preprocessing is necessary because of the poor contrast of frames in terms of inconsistencies, irregular boundaries, and objects. Filters can be used to reduce the amount of noise in a recording. The grayscale images from COVID-19 are then smoothed. Segmentation is the process of removing a specific region of interest (ROI) from the frame sense. CNN models are trained using data from the dataset's training batch, which is then used to identify test data and the infection to which it is linked. CNN layers include dense, dropout, activation, flatten, convolution2D, and MaxPool2D. An image of a patient's COVID can be used to train the software to recognise the disease. After successful training and preprocessing, the test results and the model are compared to predict infection.

### 3.4. Conv2d

To start 2D conversion, the kernel, which is a small weight matrix, is used. This kernel cuts 2D input data, performs an intelligent duplicate of a feature with the current input piece, and combines the results into a single output pixel. The kernel continues the process of each point that tilts over it, converting the 2D element matrix into another 2D feature matrix. The output elements are actually the weighted figures of the input elements (weights are the kernel values) that are placed approximately the same as the output pixel in the input layer.

### 3.5. MaxPooling2D Layer

Find the maximum value for each input channel per input window to reduce the input according to its area size (length and width) (size determined by pool size). Each window's size is gradually increased.

### 3.6. Flatten Layer

The input is flattened using the flatten command. If flatten is applied to a layer with an input shape of (batch size, 2, 2), the layer's output shape will be (batch size, 4). As a value, it accepts either channels last or channels first. The default is channels last, which recognises the input shape as (batch size, ⋯, channels), but channels first recognises the input shape as (batch size, channels, ⋯).

### 3.7. Dense Layer

Dense functionality is as follows:

(1) $$\begin{array}{c} \text{Output}=\text{activation}\left(\text{dot}\left(\text{dot},\text{kernel}\right)+\text{bias}\right), \end{array}$$

where functionality is an intelligent activation function provided as an opening parameter, kernel is a layer weight matrix, and bias is a bias layer vector (only works if bias usage is true). In addition, once a layer has been called, its features cannot be changed. Keras will generate an input layer to insert before the current layer if a popular kwarg input shape is given. This can be regarded as the same as defining an input layer directly.

### 3.8. Dropout Layer

The dropout layer, which helps to reduce overload, sets the input units to 0 anywhere at the average value per step during the training period. Input not set to 0 is increased by 1/(1 − average) so that the total amount does not change.

### 3.9. Training Process

Data from the train dataset directory is generated using the function train datagen flow from the directory. Target size specifies the final picture size. In order to generate test data for the model, you may use test datagen flow from the directory. For the training data, a fit generator is utilised, and the number of epochs defines how many times the model will run.

## 4. Experimentation Results and Analysis

The preprocessing image data generator function must be used to import our data into Keras. To produce the following picture attributes: rescale, range, zoom range, and horizontal flip, this function will also be used. A data processing tool is then used to process the images. Everything we need for our training, testing, and validation can be found in this section of the document. Using CNN as a foundation, we will build our own network from the ground up. To download the dataset used in this study, click on the following links: https://www.kaggle.com/mohammadrahimzadeh/covidctset-a-large-covid19-ct-scans-dataset and https://mosmed.ai/datasets/covid19_1110. Figures 2–4 depict the sample images from the dataset.

VGG19 and ResNet152V2 and their optimized models were used in the experiments. The accuracy, *F*-score, and receiver operating characteristic (ROC) curves have been used to evaluate the performance of our optimized models. Figures 5 and 6 show that the proposed diagnosis framework's *F*-score and accuracy increase by 1.3 percent with our optimized models. The VGG19-ResNet152V2 diagnostic framework has a 99.1 percent success rate. Our VGG19-ResNet152V2 method benefits from these enhancements because we are able to extract better features as a result. It is possible for the proposed architecture to properly understand the input graphs because of proper preprocessing measures taken. A low loss is achieved from the start, and training can be completed within a maximum of 10 epochs.

Figure 7 shows the ROC curves of the VGG19-ResNet152V2 method, which was optimized. While ResNet152V2 had the best false negative rate, VGG19 had the lowest false positive rate. Optimized VGG19, on the other hand, had the best results in terms of predicted value and F1. On the right, you can see how many epochs the implemented models are accurate over time in Figure 8. The performance of ResNet152V2 was the least stable and the most unsatisfactory of all the models tested. Pretrained models such as optimized VGG19 and ResNet152V2 consistently produced smooth results from the start and had nearly the highest accuracy of all the other research, according to our results. Optimized VGG19 and ResNet152V2 have shown smooth accuracy per epoch in this study when compared to other articles. Optimized VGG19 and ResNet152V2 *F*-score was 98.2% and 97.2% for COVID-19 images, 98.3% and 97.2% for pneumonia images, and 99.1% and 99.1% for normal images, respectively. COVID-19 images, 98.2% and 96.8% of pneumonia images, and 98.8% and 98% of normal images were correctly identified by the optimized VGG19 and ResNet152V2.

## 5. Conclusion and Future Work

Pretrained deep learning models were used in this study; both models were completely customized. Versions of the VGG19 and ResNet152V2 models were pretrained and fine-tuned. The accuracy of the paper and the models in this category were virtually identical. The collection includes 2700 COVID-19 images and 6250 pneumonia CT images. Customized deep learning models outperform the pretrained models with 96% accuracy. There will be more pretrained models and a larger dataset in future studies. These models have performed exceptionally well in terms of our dataset. An outstanding performance has been achieved by the optimized VGG19 and the ResNet152V2 in this context. Edges could be recognised from original photos or feature maps using just six layers that included ReLU activation, drop operation, and maximum pooling. With an accuracy rate of 98%, our model outperforms the current CNN models. Numerous evaluations of various parameter metrics proved the efficacy of our proposed approach. Using these models, CT scans can detect COVID-19 and pneumonia quickly. As a result, COVID-19 and pneumonia can be detected with relative ease using this method. As a result of this method, the virus can be tested and tracked quickly without the risk of getting caught in a line and spreading the virus. As a result of this discovery, the medical community will never be the same again. COVID-19 and pneumonia patients using this method are to blame for the current pandemic. Deep learning-based COVID-19 detection methods may be especially useful in light of the large number of patients who are at risk.

## Figures and Tables

**Figure 1:** Proposed VGG19-ResNet CNN architecture.

**Figure 2:** Normal images.

**Figure 3:** Pneumonia images.

**Figure 4:** COVID-19 images.

**Figure 5:** *F*-score comparison analysis.

**Figure 6:** Accuracy comparison analysis.

**Figure 7:** ROC curve: combined VGG19 and ResNet152V2.

**Figure 8:** Epoch comparison.

**Table 1:** Related work comparison.

Reference	Method	Commonalities	Differences
[22]	Generative adversarial networks (GANs), extreme learning machine (ELM), and long/short term memory (LSTM)	Pretrained architectures were used	Geographical issues were considered
[18]	Review study	Statistical models are explained	Robustness and reliability of statistical models are compared
[23]	Deep neural network	Conceptual deep learning framework developed	Drug development benefits explained
[24]	Review study	Statistical models are explained	Deep Boltzmann machines (DBM), restricted Boltzmann machine (RBM), deep belief network (DBN), Hopfield network, and long-short-term memory (LSTM) were explained

**Table 2:** Model layers.

Layer	Output shape	Parameters
resnet152v2	4,4,2048	52,442,528
reshape_3	4,4,2048	0
flatten_3	98776	0
dense_3	512	32742678
dropout_2	512	0
dense_3	1	254

## Data Availability

The data used to support the findings of this study are included within the article.

## Abbreviations

AI: Artificial intelligence
ARDS: Acute respiratory distress syndrome
CNN: Convolutional neural network
CT: Computed tomography
DBM: Deep Boltzmann machines
DBN: Deep belief network
DL: Deep learning
ELM: Extreme learning machine
GAN: Generative adversarial networks
LSTM: Long/short term memory
ML: Machine learning
RT-PCR: Reverse transcription polymerase chain reaction
RBM: Restricted Boltzmann machine
ReLU: Rectified linear unit
ROC: Receiver operating characteristic
ROI: Region of interest
VGG: Visual geometry group.
